RETRACTED

# Comparison of traditional and new generation DNA markers declares high genetic diversity and differentiated population structure of wild almond species

**DOI:** 10.1038/s41598-017-06084-4

**Published:** 2017-07-20

**Authors:** Karim Sorkheh, Mehrana Koohi Dehkordi, Sezai Ercisli, Attila Hegedus, Júlia Halász

**Affiliations:** 1 Department of Agronomy and Plant Breeding, Faculty of Agriculture, Shahid Chamran University of Ahvaz, P.O. Box 61355/144 Ahvaz, Iran; 2 Department of Agronomy, Faculty of Agriculture, Payame-Noor University, P.O. Box 19395-3697 Tehran, Iran; 3 Department of Horticulture, Agricultural Faculty, Ataturk University, 25240 Erzurum, Turkey; 4 Department of Genetics and Plant Breeding, Szent István University, H-1118 Budapest, Villányiút 29–43 Hungary

## Abstract

Wild almond species as sources of genetic variation may have crucial importance in breeding. A total of 389 accessions of 18 species have been analysed using inter-retrotransposon amplified polymorphism (IRAP), retrotransposon-microsatellite amplified polymorphism (REMAP), sequence-specific amplification polymorphism (S-SAP), amplified fragment length polymorphism (AFLP), inter simple sequence repeat (ISSR) and simple sequence repeats (SSR). Retrotransposon markers indicated the presence and movement of some Ty3-*gypsy* and Ty1-*copia*-elements in almond genome. Since transposable elements are associated with large-scale genome alterations, REMAP produced more reliable phylogenetic inferences than AFLP where homoplasy may affect clustering. In addition, high resolution melting (HRM) analysis was developed to detect SNPs. HRM analysis revealed 1:189 bp frequency of SNPs in exon positions, and the transition-to-transversion proportion was 1.84:1. The low transition bias suggests low methylation levels in almond genome. The polymorphic information content (PIC) was the highest for SSR markers, while SNPs had an average PIC of 0.59, which is close to the values of the rest of the markers. Huge genetic diversity, fragmented population structure and footprints of human selection was confirmed by merging information from all marker strategies. Considering time, cost and performance HRM can be a marker of choice in future studies of *Prunus* diversity.

## Introduction

To promote crop improvement, it is crucial to be aware of the genetic diversity and relatedness in the breeding material. Wild almond species demonstrate high resistance to biotic and abiotic stress as well as provide valuable germplasm resources for satisfactory breeding^1^. Controlled hybridization and selection programs are implemented to favourad vantageous traits in diverse ways, but it may also result in the loss of genetic diversity in most annual species^2^; this is particularly evident in out breeding species including almond and related *Prunus* species (*Prunus* spp. L.)^3^.

RETRACTED

Wild species are important sources of genetic diversity if they can be crossed with crop plants^4^. Secondary and tertiary gene pools of crop plants may also consist of numerous closely related species. Almond is native to Central Asia and many related species grow in the near east region^5^. Sorkheh *et al*.^6^ investigated the phenotypic diversity, distribution and morphological characterization of Iranian wild almond species, but there are very few studies related to the ecology and population structure of wild almond species. Description of such resources is important in order to identify areas of diversity, to utilize them as almond genetic resources in conservation and breeding.

Due to various distributions and evolutionary histories, there are many different wild relatives of crops. In species complexes related to crops, a number of clades may have occupied original regions fairly recently, for example after the last glacial period, and migration bottlenecks were also possible over this time^7^. These processes are inadequately understood in the majority of non-domesticated plants, although they may have a crucial impact on the conservation/breeding programs exploiting wild relatives. Introgression may serve as a bridge in the spatial variation in wild resources and cultivated genotypes. Finally, inherent diversity in non-cultivated species are adapted to specific environmental conditions, which might be utilized through introgression in crops^8^.

Knowledge on genetic diversity and relatedness is important to design strategies for preservation, as well as organizing accessions of wild species with appropriate attributes, designed for use as breeding material. Therefore, molecular characterization has become the most important tool for evaluating genetic diversity and similarity within and between populations or accessions, mapping of functional genes, assembly of genetic linkage maps, marker-assisted selection (MAS), and phylogenetic experiments in crop species^9^.

In addition, several molecular marker techniques based on retrotransposons (RTNs) have been developed^10–12^. Distributions of RTNs in plant genomes provides the basis for developing marker systems, and compare them with other markers RTN markers seem to be useful and polymorphic in many species^13^. The need for RTN sequence information is a major limitation to design family-specific primers. A number of studies have demonstrated that due to homology, RTN sequences between long terminal repeat (LTR)-RTN plant families can be used across species^14, 15^.

RETRACTED

Evaluation of genetic diversity of the genus *Medicago* using Tms1Ret1 LTR-based sequence-specific amplification polymorphism (S-SAP) had a high marker index for S-SAP compared to amplified fragment length polymorphism (AFLP) and selective amplification of microsatellite polymorphic loci (SAMPL)^16^. Conversely, S-SAP relies on digestion and the sensitivity to DNA methylation of generally-used enzymes, for example, *Pst*I and *EcoR*I, is associated with the variable degree of CG and CXG methylation in plant DNA^17^, which means that a number of evident polymorphisms could be neither sequence-based nor heritable. Inter-retrotransposon amplified polymorphism (IRAP) and retrotransposon-microsatellite amplified polymorphism (REMAP) are two RTN-based markers that do not require DNA digestion and can be used in genetic differentiation^12, 13, 18^.

Due to a high degree of polymorphisms, simple-sequence repeats (SSRs) have been recognized as valuable markers in plants and animals, and therefore the majority of genetic studies in *Prunus* species have usually been based on SSR markers^19–21^. Although the majority of these SSRs have been developed in peach^22^, it has been established in numerous studies that these markers were robust in other *Prunus* species such as cherry, almond, or plum^21, 22^. On the other hand, an important drawback of SSR analysis is the elevated price of the fluorescent labels. Conversely, SNP markers are present in large quantities in the plant genome^23^ and thus can be used as genetic markers for cultivar recognition, assembly of genetic maps, measurement of genetic diversity, or marker-assisted breeding^24, 25^. In addition, the recognition of SNPs and INDELs has been simplified by the current progress in sequencing technology. HRM analysis was developed to identify SNPs in PCR amplicons as it is a simple and low-cost method^25^. Recently, this advance has been used for genetic mapping^24, 26^. HRM was also used to check mutation in large multi-exon genes to discover disease-related alterations in humans^26^ and construct linkage maps in crop species^24^. Wu *et al*.^25^ used HRM analysis to detect SNPs in EST sequences that have been retrieved from a database.

This study was carried out to evaluate the usefulness of formerly published (REMAP, IRAP and S-SAP) and newly designed (IRAP and REMAP) RTN-based markers compared to formerly published (ISSR, SSR, EST-SSR and AFLP) and newly designed (EST-SSR) non-RTN-based markers for the discrimination and phylogenetic analysis of *Prunus* species. In addition, the current investigation applied the HRM approach to identify SNPs in wild almond species based on publicly available *Prunus* ESTs and next generation sequencing (NGS) data, and established a technique for SNP detection and genotyping to characterize genetic variation in wild species that might be exploited in almond breeding programs. Data were also informative on demographic and evolutionary history of species that are close relatives of a long cultivated crop plant.

RETRACTED

## Results

### RTN activity in wild almond species and IRAP analysis

To analyse genetic variations in 389 individuals of 18 wild almond species (Table 1) a total of 22 single, and 60 IRAP primer combinations (Table 2) from *Prunus* and non-*Prunus* RTN families were used. All single IRAP primers (designed based on Sukkula, Daniela, Fatima and RTNs LORE1 and LORE2) generated discernible and polymorphic banding patterns (a representative banding pattern is shown in Fig. S1). Single IRAP primers (designed based on RTN Tps12a from *Pisum sativum*) also amplified scorable but not polymorphic banding patterns. IRAP amplification of RTNTps19 (from pea), showed a non-scorable banding pattern at low annealing temperature (less than 40 °C) (results not shown).

**Table 1:** Wild almond species populations used in this study, and their origin.

Section	Species	No of accessions	Geographical origin	Abb. pop.
Euamygdalus	*P. carduchorum*	21	Piranshahr	CAR
	*P. communis*	22	Shahrekord	COM
	*P. elaeagnifolia*	23	Bazoft	ELA
	*P. fenzliana*	25	Marand	FEN
	*P. korschinskyi*	22	Oroomieh	KOR
	*P. kotschyi*	21	Shiraz	KOT
	*P. orientalis*	20	Kareh-e Base	ORI
	*P. trichamygdalus*	24	Sardasht	TRI
Lycioides	*P. eburnea*	21	Baneh	EBU
	*P. erioclada*	20	Shiraz	ERI
	*P. lycioides*	18	Lordegan	LYC
	*P. reuteri*	19	Lordegan	REU
	*P. urumiensis*	22	Oroomieh	URU
Spartioides	*P. arabica*	20	Felard	ARA
	*P. glauca*	19	Lordegan	GLA
	*P. haussknechtii*	24	Koohrang	HAU
	*P. pabotii*	20	Mahabad	PAB
	*P. scoparia*	27	Saman	SCO
***Total***		***389***

**Table 2:** IRAP and REMAP primer combinations used in this study.

Primer	Annealing temp. (°C)	Loci			He	Ne	I	Band size (bp)
IRAP		Total	Polymorphic	% polymorphic				
Sukkula LTR1	59	15	12	80	0.36	1.44	0.38	75–1500
Wilma-Bagy2	60	19	19	100	0.31	1.48	0.41	300–2000
Daniela LTR2	60	20	12	60	0.24	1.74	0.55	400–1500
Fatima LTR	60	14	13	92.8	0.30	1.57	0.41	300–2000
5LTR-Sukkula LTR1	61	16	15	93.7	0.33	1.65	0.48	200–1300
5LTR-Daniela LTR1	61	12	12	100	0.35	1.43	0.47	200–700
Bare1 LTR-Sukkula LTR1	60	10	10	100	0.23	1.43	0.47	200–1500
Bare1 LTR-Daniela LTR2	60	13	12	92.3	0.28	1.55	0.33	100–1500
Bare1 LTR-Sukkula LTR2	63	18	16	88.8	0.34	1.63	0.47	200–2000
Tms1Ret1	63	12	9	75	0.30	1.45	0.41	100–1500
LORE1	58	11	8	72.7	0.29	1.33	0.42	200–1500
LORE2	55	9	6	66.7	0.24	1.54	0.48	200–1500
Tps12a	54	4	1	25	0.23	1.44	0.38	200–700
Tms1Ret1- LORE1	61	5	3	60	0.22	1.23	0.45	200–1000
Tms1Ret1- LORE2	60	12	10	83.3	0.30	1.32	0.55	300–1500
Tms1Ret1- Tps12a	58	13	8	61.5	0.32	1.35	0.44	300–1500
LORE1-LORE2	58	9	6	66.7	0.25	1.38	0.46	300–1500
LORE1-Tps12a	59	6	4	66.7	0.24	1.37	0.42	420–1500
LORE2-Tps12a	56	7	1	14.2	0.20	1.34	0.38	800–15000
REMAP								
WIS2–1A LTR-UBC815	63	12	12	100	0.41	1.70	0.59	400–1500
Sukkula LTR1-UBC815	57	15	13	86.7	0.35	1.69	0.54	100–1500
Wilma-Bagy2-UBC815	63	18	15	83.3	0.39	1.74	0.62	300–1500
Daniela LTR1-UBC815	58	12	10	83.3	0.43	1.32	0.54	200–2000
Daniela LTR2-UBC815	62	11	10	90.9	0.38	1.50	0.26	500–2000
Fatima LTR-UBC815	58	18	16	88.8	0.45	1.33	0.36	300–2000
Wis LTR2-UBC818	58	17	12	70.5	0.21	1.47	0.48	75–1500
Sukkula LTR1-UBC825	60	16	14	87.5	0.30	1.25	0.62	200–2000
Wilma-Bagy2-UBC840	60	12	11	91.7	0.40	1.58	0.58	300–2000
Daniela LTR1-UBC840	60	15	13	86.7	0.38	1.65	0.45	200–2000
Wis LTR2-UBC848	57	16	15	93.7	0.32	1.50	0.53	300–1500
WIS2–1A LTR-UBC857	58	14	14	100	0.40	1.69	0.62	200–2000
Sukkula LTR1-UBC857	60	12	12	100	0.39	1.48	0.64	100–1500
Wis LTR1-UBC857	58.9	13	11	84.6	0.34	1.47	0.58	300–1500
Wis LTR2-UBC857	59.4	10	9	90	0.32	1.54	0.62	300–1500
Daniela LTR1-UBC857	60.7	12	5	41.6	0.21	1.35	0.54	200–1500
Daniela LTR2-UBC857	58.3	11	8	72.7	0.25	1.44	0.58	200–1500
Wis LTR1-A13	58	18	17	94.4	0.36	1.65	0.49	300–1500
Wilma-Bagy2-A13	62	15	15	100	0.38	1.80	0.53	200–1500
Daniela LTR1-A13	62	11	11	100	0.39	1.78	0.53	300–1500
Tms1Ret1–459	52	14	11	78.5	0.44	1.33	0.48	500–2500
Tms1Ret1-A7	52	5	1	20	0.38	1.45	0.34	350–850
Tms1Ret1-A12	52	12	6	50	0.35	1.41	0.47	700
Tms1Ret1-B1	52	2	1	50	0.34	1.32	0.38	200–1000
Tms1Ret1–438	51	8	5	62.5	0.41	1.23	0.39	500–1000
Tms1Ret1–443	52	5	2	40	0.38	1.48	0.42	150–700
Tms1Ret1–818	52	6	3	50	0.39	1.55	0.41	200–1000
Tms1Ret1–825	52	9	4	44.4	0.41	1.35	0.42	200–850
LORE1–840	52	8	2	25	0.36	1.74	0.52	200–1000
LORE1–848	52	7	3	42.8	0.38	1.65	0.51	200–1400
LORE2–849	52	9	3	33.3	0.42	1.55	0.42	350–1000
LORE2–857	52	12	5	41.6	0.32	1.30	1.38	500–1000
Tps12a-459	52	9	7	77.7	0.33	1.25	1.23	300–1000
Tps12a-438	52	7	4	57.1	0.40	1.45	0.35	200–1500

IRAP primer combinations of RTN families of *Prunus* and other origins created polymorphic and scorable banding patterns, except the primer Tps19. Ten out of the 19 IRAP primers produced 225 loci. Of these 225 amplified loci, 157 were polymorphic (69.9%). The primer combination Bare 1LTR- Sukkula amplified the most polymorphic loci. The average number of polymorphic loci was 9.32 per primer. The size of the amplified IRAP loci ranged from 75 to 2,000 bp (Table 2).

RETRACTED

IRAP-based UPGMA dendrogram grouped populations into three major groups (Fig. 1). Group I integrated populations CAR, COM, ELA, FEN, KOR, ORI and TRI. The second group included REU, GLA, HAU, PAB and SCO (abbreviations of populations are explained in Table 1). Populations from the Lyciodes section were found in the third group. Similarly to the results of the cluster analysis, the populations EBU, ERI, URU, ARA, and LYE were distinct from the rest of the population on PCA biplot derived from IRAP markers (data not shown). To evaluate and partition the total genetic variation between and within populations, AMOVA was carried out based on the eight populations using IRAP data. Significant differences (*P* < 0.05) were evident within populations. The level of genetic variation was higher between populations (80%) compared to within populations (20%). The characteristics of amplified IRAP loci using 19 primers are displayed in Table 3. The percentage values of IRAP polymorphic loci in population ranged from 47.6 (FEN) to 89.6 (KOT), with an average of 80.44. The frequency of all IRAP amplified loci was greater than 5%. A genotype-specific locus was generated in the population CAR by IRAP primer combination Tms1Ret1-LORE1. Primer LORE2 amplified a specific locus in a genotype of population EBU. Mean heterozygosity varied from 0.208 (ORI and SCO) to 0.261 (CAR), averaging 0.234 (Supplementary Table S1).

**Figure 1:** Dendrogram obtained with the similarity simple matching (SM) coefficient pair group method with the arithmetical average clustering algorithm from 289 IRAP markers for 389 wild almond species. The value on the dendrogram gives the stability of nodes estimated with a bootstrap procedure (no number indicates support less than 10%). Bar graphs showing genetic diversity structure for the 389accessions of *Prunus* species as assessed using STRUCTURE software. Each group is represented by a different color (blue, red and green).

**Table 3:** Characteristics of amplified IRAP, REMAP and IRAP + REMAP loci in studied wild almond species populations.

Population	CAR	COM	ELA	FEN	KOR	KOT	ORI	TRI	EBU	ERI	LYC	REU	URU	ARA	GLA	HAU	PAB	SCO
**IRAP**																		
Number of loci	61	58	55	64	48	53	56	64	50	47	49	68	66	42	41	53	56	60
Percentage of polymorphic loci (%)	87.4	78.79	88.42	47.65	89.40	89.6	74.3	80.6	83.6	77.5	87.5	68.8	88.9	89.4	87.4	82.3	74.6	71.8
Number of loci with frequency ≥5%	61	58	55	64	48	53	56	64	50	47	49	68	66	42	41	53	56	60
Number of private loci	1	0	0	0	0	0	0	0	1	0	1	0	0	0	0	0	0	0
Number of less common loci (≤25%)	0	0	1	0	1	0	0	0	0	0	0	1	1	1	0	1	0	0
Number of less common loci (≤50%)	5	3	3	5	0	0	2	3	5	4	0	0	0	0	0	5	3	3
Mean of heterozygosity	0.26	0.23	0.23	0.26	0.25	0.25	0.208	0.22	0.22	0.22	0.24	0.24	0.24	0.25	0.23	0.25	0.22	0.208
Standard error of mean heterozygosity	0.02	0.02	0.02	0.02	0.02	0.02	0.02	0.02	0.20	0.02	0.02	0.02	0.02	0.02	0.02	0.02	0.02	0.02
**REMAP**																		
Number of loci	50	54	50	55	56	54	60	62	48	49	65	42	50	53	41	56	49	60
Percentage of polymorphic loci (%)	81.2	85.2	80.64	85.32	88.64	63.24	72.35	83.25	75.65	68.25	84.32	65.89	88.25	74.65	87.35	85.69	75.65	74.32
Number of loci with frequency ≥5%	50	54	50	55	56	54	60	62	48	49	65	42	50	53	41	56	49	60
Number of private loci	0	0	0	0	1	1	0	1	0	1	0	0	1	1	0	1	1	1
Number of less common loci (≤25%)	0	2	0	0	0	0	0	0	0	0	0	0	0	0	0	0	0	0
Number of less common loci (≤50%)	0	3	1	1	1	1	1	1	1	1	1	1	1	0	0	0	0	0
Mean of heterozygosity	0.26	0.25	0.27	0.28	0.26	0.25	0.25	0.325	0.26	0.24	0.25	0.27	0.24	0.25	0.23	0.22	0.23	0.20
Standard error of mean heterozygosity	0.02	0.02	0.02	0.02	0.02	0.02	0.02	0.023	0.02	0.02	0.02	0.02	0.02	0.02	0.02	0.02	0.02	0.02
**IRAP** **+** **REMAP**																		
Number of loci	111	112	105	119	100	107	116	126	98	96	114	110	116	95	82	109	105	120
Percentage of polymorphic loci (%)	82.6	83.2	86.2	82.5	79.6	81.2	80.3	78.5	84.2	82.7	80.2	79.6	82.4	79.2	83.2	86.3	79.7	82.1
Number of loci with frequency ≥5%	111	112	105	119	100	107	116	126	98	96	114	110	116	95	82	109	105	120
Number of private loci	1	0	0	0	1	1	0	1	1	1	1	0	1	1	0	1	1	1
Number of less common loci (≤25%)	0	2	1	0	1	0	0	0	0	0	0	1	1	0	0	1	0	0
Number of less common loci (≤50%)	5	6	4	6	1	1	3	4	6	5	1	1	1	1	0	5	3	3
Mean of heterozygosity	0.26	0.24	0.25	0.27	0.26	0.25	0.23	0.27	0.24	0.22	0.25	0.25	0.24	0.25	0.23	0.23	0.23	0.21
Standard error of mean heterozygosity	0.01	0.01	0.02	0.02	0.02	0.01	0.01	0.02	0.02	0.02	0.02	0.02	0.01	0.01	0.01	0.02	0.02	0.02

RETRACTED

### REMAP analysis

Of the 48 REMAP primer combinations investigated, 34 produced 391scorable bands. The primer combination Tms1Ret1-A7 created a monomorphic banding pattern. No bands were amplified using REMAP primer combinations with RTN Tps19. Of the391 amplified bands, 300 were polymorphic (71.2%) (a representative banding pattern is shown in Fig. S2). The average number of polymorphic bands was 8.82 per primer. The size of the amplified fragments varied from 100 to 2,500 bp.

There were three well-known important clusters, based on REMAP data (Fig. 2). Group I consisted of two subgroups: CAR, COM, ELA, FEN, KOR and KOT in subgroup I, and ORI and TRI in subgroup II; the species belonging to the Lycioides section were grouped in group II. The third group consisted of the populations REU, GLA, HAU, PAB, and SCO. Associations between 18 populations using REMAP markers were well-established through PCA (data not shown). REMAP-based AMOVA was approved using the 18 populations for the basis of the analysis. Similar to the results acquired by the IRAP method, the level of genetic variation was higher between populations (92%) compared to within populations (8%), demonstrating clear discrimination of the studied populations. The characteristics of amplified loci by means of 34 REMAP primers are shown in Supplementary Table S1.

RETRACTED

**Figure 2:** Dendrogram obtained with the similarity simple matching (SM) coefficient pair group method with the arithmetical average clustering algorithm from 587 REAMP markers for 389 wild almond species. The value on the dendrogram gives the stability of nodes estimated with a bootstrap procedure (no number indicates support less than 10%). Bar graphs showing genetic diversity structure for the 389accessions of *Prunus* species as assessed using STRUCTURE software. Each group is represented by a different color (blue, red and green).

The percentage of polymorphic loci in a population based on REMAP data varied from 63.2 (KOT) to 88.6 (KOR), with an average value of 78.9. Two loci with a frequency of less than 25% were detected (Supplementary Table S1), suggesting that most of the amplified loci are common in the studied populations. Nine genotype-specific REMAP loci were identified in populations KOR, KOT, TRI, ERI, URU, ARA, HAV, PAB and SCO. The mean of heterozygosity varied from 0.221 (HAU) to 0.275 (FEN), with an average of 0.267.

### Combined data IRAP and REMAP analysis

The combined data of IRAP and REMAP markers were utilized to construct a dendrogram to calculate the influence of both techniques when taken together. Populations were assembled into three most important clusters (Fig. 3). Group I included COR, COM, ELA, KOR, KOT, ORI and TRI. Populations EBU, ERI, URU, ARA and LYC clustered in group II and REU, GLA, HCU, PAB, and SCO were classified into group III. A PCA of the IRAP + REMAP data was used to validate associations between eighteen populations.

**Figure 3:** Dendrogram obtained with the similarity simple matching (SM) coefficient pair group method with the arithmetical average clustering algorithm from 876 IRAP + REAMP markers for 389 wild almond species. The value on the dendrogram gives the stability of nodes estimated with a bootstrap procedure (no number indicates support less than 10%). Bar graphs showing genetic diversity structure for the 389accessions of *Prunus* species as assessed using STRUCTURE software. Each group is represented by a different color (blue, red and green).

The first (PCA1) and second (PCA2) principle coordinates accounted for 33% and 21% of the total variation, respectively. Relationships between populations on the biplot were similar to the results acquired from cluster analysis. AMOVA was carried out to investigate total genetic variation between and within populations. Similar to that shown by IRAP and REMAP markers, the level of genetic variation was higher between populations (83%) compared to within populations (7%). The percentage of polymorphic loci in populations varied from 78.5 (TRI) to 86.35 (HAU), with an average of 81.9. The mean of heterozygosity varied from 0.206 (SCO) to 0.272 (TRI), with an average of 0.242 (Supplementary Table S1). Due to high genetic diversity between populations, IRAP + REMAP-based cluster analysis was carried out using complete linkage algorithms based on simple matching (SM) similarity coefficient to recognize groups among all 389 wild almond accessions.

RETRACTED

### SSR and EST-SSR for fingerprinting *Prunus* spp

As there is a lack of a standardized set of microsatellite primers for almond, primer pairs of closely related species have been regularly used in molecular descriptions^27–29^. In this study, amplification of genomic DNA was performed for 219 SSR and EST-SSR loci designed from different *Prunus* species (peach, almond, plum, sweet cherry, and sour cherry). For every examined locus, calculated indices are shown in Supplementary Table S2.

Data of nine primer pairs with either in distinguishable amplification (PS01H03, EPPISF027, UDP96-001, CPDCT027, BPPCT025, and CPPCT006), stutter bands (UDP96-019), or monomorphic bands (EPPISF014 and EPPISF025) were excluded from the analysis. The rest of the 210 primer pairs provided clear and polymorphic multi-allele bands for all accessions of almond and related *Prunus* samples.

The total number of examined alleles (na) was 16,948, ranging from 50 to 90, with an average of 81.1 alleles per locus. SSR primers derived from the non-coding DNA region had more alleles (17,141 alleles) than EST-SSR primers (14,189 alleles). The average number of alleles per locus were similar in both types of SSRs (80.8 and 81.1 alleles per locus for SSR and EST-SSR, respectively). PruAvest-3, PruMest-5, Prupest-2 and PruPest-36 had the highest number of alleles (90).

The number of effective alleles (ne) was 5,512.15, with a maximum of 43.84 in BPPCT039, PruArest-2, PruAvest-10, Prumest-6, PruCest-1, PruPest-25, Prupest-53 and PruPest-81, and a minimum of 9.69 in EPPISF018, PruAvest-6, PruMest-2, PruDest-3, PruPest-23, PruPest-49 and PruPest-77 loci. Loci with a higher number of effective alleles were more powerful in discriminating genotypes.

The average frequency of the major allele was 0.36, with a maximum of 1.10 in EPPISF018 and a minimum of 0.25 in the BPPCT039, PruArest-4, PruAvest-4, PruAvest-24, PruMest-12, PruDest-5, PruPest-15, PruPest-35, PruPest-55 and PruPest-75loci. The high allelic diversity of microsatellite loci revealed high genetic variation in the wild almond germplasm investigated in this study. The sizes of the amplified DNA fragments of all the loci ranged from 70 to 508 bp. The smallest DNA fragment (70 bp) amplified was in an accession of *P. scoparia* (accession number #350) in locus UDP98-412. Allele sizes in this locus ranged from 70 bp in *P. scoparia* (accession number #350) to 191 bp in *P. orientalis* (accession number #130), which was generally lower compared to other loci. The largest allele, 508 bp, was found in the pchgms5 locus in the accession of wild almond species of *P. elaeagnifolia* (accession number #66). The locus pchgms5 amplified a diverse range of alleles for different groups of accessions. The allele sizes of this locus ranged from 429 to 508 bp in cultivated almond and some related species (*P. orientalis*, *P. spartioides*, and *P. lycioides*), while in *P. chameamygdalus*, *P. leptopus*, peach and plum, the size of the amplified alleles was 139–162 bp. The greater difference in the size of the amplified alleles was related to the presence of most divergent samples (from different locations and species) used in this experiment.

RETRACTED

Expected heterozygosity across the tested loci ranged from 0.18 in EPPISF018 to 0.98 in BPPCT039, PruArest-7, PruAvest-12, PruMest-5, PruDest-3, PruPest-18, PruPest-43 and PruPest-68, with an average of 0.91. The range of expected heterozygosity of the selected species in this work was greater than that reported previously. Observed heterozygosity ranged from 0.09 in EPPISF001 to 0.80 in CPPCT005, PruArest-9, PruAvest-13, PruMest-5, PruDest-2, PruPest-16, pruPest-40, Prupest-64, with an average of 0.60. In all loci, the expected heterozygosity was higher than the observed heterozygosity, implying allele fixation in the studied loci.

The mean value of the fixation Index (Fis) was 0.183, indicating the excess heterozygosity between samples. The average total inbreeding coefficient (Fit) was 0.406, with a maximum of 0.7912 in EPPISF001, and a minimum of 0.133 in CPPCT002, PruArest-11, PruAvest-14, PruMest-5, PruDest-1, PruPest-14, PruPest-37, PruPest-60 and PruPest-83. In this study, null alleles were found in some loci, which may partly account for the lower percentage of heterozygosity. The average gene flow index (Nm) was 0.721, and values ranged from 0.313 in EPPISF011 to 1.295 in CPSCT012, PruArest-18, PruAvest-21, PruMest-12, PruCest-2, PruPest-21, PruPest-44 and PruPest-67. It demonstrates a comparatively low level of genetic material exchange (seed, pollen etc.) between assumed populations.

RETRACTED

Gene diversity between the loci varied from a minimum of 0.183 to a maximum of 0.977, with an average of 0.903 (Supplementary Table S2). The mean value of polymorphism information content (PIC) was 0.912, with a minimum of 0.170 in EPPISF018, and a maximum of 0.971 in BPPCT032, PruArest-5, PruAvest-8, PruAvest-30, PruMest-22, PruPest-31, PruPest-54 and PruPest-77 loci.

In germplasm studies, the PIC was greater in the EST-SSR loci (0.919) than in the SSR loci (0.874), which showed that EST-SSR markers were more suitable than SSRs for recognizing genetic variation. The 174 EST-SSRs used in this experiment were developed from the *Prunus* genus. They had a range of polymorphism (PIC = 0.699–0.971) in the samples studied.

Shannon’s information index (I) demonstrated high correlation (*r* ^2^ = 0.96) with PIC values. The average Shannon index was 4.116, ranging from 1.356 in EPPISF018 to 4.679 in BPPCT039, PruArest-6, PruAvest-9, PruAvest-32, PruMest-23, PruPest-9, PruPest-32, PruPest-55 and PruPest-78 loci. The proportion of homozygous loci was under 25% for the majority of the accessions (Supplementary Table S2) and the average number of homozygous loci was 45. Cross-pollination, mainly due to self-incompatibility, results in low level of homozygosity. The lowest levels of homozygosity were observed in *P. argentea* and *P. trichamygdalus*.

### SNP identification and detection from EST and RNA-seq databases

All EST (111,699) sequences of *Prunus* species, namely peach (*P. persica*; 80,797), apricot (*P. armeniaca*; 15,105), sweet cherry (*P. avium*; 6,035), Japanese apricot (*P. mume*; 4,589), almond (*P. dulcis*; 3,864), sour cherry (*P. cerasus*; 1,255) and European plum (*P. domestica*; 54) were downloaded from GenBank (ftp://ncbi.nlm.nih.gov/genbank/genomes/). To construct longer and less redundant sequences, publicly-available ESTs were assembled from CAP3. CAP3 is a commonly used program^29^ that identifies overlapping sequences and creates contigs with consensus sequences. A total of 111,699 *Prunus* EST sequences were brought together into 12,159contigs, and 125 EST contigs were predicted to have SNPs with a redundancy score ≥2 according to Wu *et al*.^25^, and adequate flanking sequences for primer design. In addition, 100 EST contigs with putative SNPs were chosen from a *Prunus* SNP database at ESTree for HRM analysis. In total, 125 EST contig sequences were used for primer design to confirm and/or recognize SNPs by HRM analysis. The sequences of the SNP primers used in the study are shown in Supplementary Table S3.

### SNP-HRM analysis and fingerprinting for genetic diversity of *Prunus* spp

Preliminary selection of a panel of 389 accessions of wild almond (*Prunus* spp. L.) species was achieved using 100 SNP markers. The allele nomenclature was based on the Tm values combined with a thorough analysis of melting peaks. The SNP primer pairs created a total of 2,315 alleles in 389 accessions ranging from 6 (including SNP4, SNP5, SNP10, SNP12, SNP15) to 11, with a mean of 8.3 alleles per locus (Supplementary Table S4). The observed heterozygosity (Ho) ranged from 0.16 to 0.68. Expected heterozygosity was generally higher, and ranged from 0.42 to 0.77. The PIC ranged from 0.403 to 0.763 with an average of 0.59. Based on PIC values, SNP31, SNP57, SNP77, SNP97, SNP117, SNP137, SNP157, SNP177, SNP197, SNP217, SNP237, SNP257 and SNP277 were the least informative, while SNP24, SNP50, SNP70, SNP90, SNP110, SNP130, SNP150, SNP170, SNP190, SNP210, SNP230, SNP250 and SNP270 were the most informative loci.

RETRACTED

Of the125 EST contigs, HRM analysis demonstrated that 100 contigs had polymorphic melting curves when assayed against the test population consisting of 389 accessions of wild almond species, while 25 were monomorphic, representing putative sequencing errors in the SNP sites of the EST, or that a common SNP allele was present in the *Prunus* species population used in the present study. The polymorphisms identified by HRM analysis incorporated SNPs, INDELs and microsatellite variations. Flanking sequence information and related GenBank accession numbers of the SNPs are available in the dbSNP database (http://www.ncbi.nlm.nih.gov/SNP/). All four classes of SNPs^25^ were identified by HRM analysis, and the genotypes with different SNP alleles were distinguished by distinct melting profiles. A/T transversions were considered to be the SNP difference most difficult to resolve by melting analysis^31, 32^.

### Genetic relatedness of the accessions of *Prunus* spp. based on SNP-HRM

A total of 389 accessions of wild almond species were genotyped using HRM analysis, and data were used for phylogenetic analysis. The results demonstrated that apanel of 17 exon fragments as well as SNPs, INDELs and a microsatellite were able to determine the genetic differences between the accessions of studied wild almond species. At the hierarchy levels, where a small group of the accessions was formed, the bootstrap values were relatively high for most of the clusters, while at higher hierarchy levels, the bootstrap values became much lower (most frequently they reached the value 100). Therefore, the tree can only consist of groups of accessions closely related. Consequently, 389 accessions of wild almond species were divided into three groups.

### Population genetic structure inference

From the outcome of population structure analysis using each marker system, we observed maximum value of ΔK at K = 2, followed by K = 3 and K = 4, while distribution of ln(K) stabilized at K = 3. Thus three genetic groups were identified in the population. Under the non-admixture model at K = 3, the three clusters (G1, G2, and G3) had a share of 40.9, 78.3, and 37.8% of the population, respectively. At K = 3, cluster 1 differentiated the wild germplasm accessions that including in Euamygdalus section. Under the admixture model, genetic admixtures was high at K = 3. At K = 3, cluster 1and cluster 2 exhibited high divergence (0.45). Cluster II differentiated the cultivars from Spartioides section and exhibited closer genetic relatedness with cluster 1. Genetic admixture was higher in the wild population. At K = 4, clear population structure differentiation could be identified. Cluster 3 included wild species from Lycioides section.

RETRACTED

On the basis of the molecular data, the results from Bayesian clustering analysis using STRUCTURE software confirmed the groupings we observed in UPGMA dendrogram and PCA. The most likely value of K (as chosen by Evanno’s DK method) in Bayesian clustering analysis was three, which indicates the division of variation into three clusters, indicating the most appropriate four main clusters within the wild *Prunus* species populations studied, confirming the clustering of UPGMA dendrogram and PCA. The first cluster (blue colour) consisted of population from Euamygdalus section. The populations from Spartioides section were placed into the second cluster (red colour), while, population of Lycioides section were placed into the third cluster (green colour).

Overall, we found an admixture model to be more effective than a non-admixture model for markers based population structure analysis. This approach identified more groups in the population for each marker (K = 3).

### Population demography inference

Results of Tajima’s D and Fu’s Fs tests for the 18 populations, Euamygdalus section, the Spartioides section, and the Lycioides section are shown in Table 4. Values of both tests were significant and negative for all three groups, suggesting a possible historical population expansion. Furthermore, mismatch distributions for the Euamygdalus, Spartioides and Lycioides sections were unimodal and supported the hypothesis of the sudden expansion model (Fig. 4). The low and non-significant raggedness index values (Table 4) suggested a significant fit between the observed and the expected distributions.

**Table 4:** Tajima’s D, Fu’s Fs and parameters of the mismatch distribution for almond populations based on all markers.

Population	Tajima’s D	Fu’s Fs	t	SSD (PSSD)	Raggedness (Pr)
CAR	−2.306**	−6.031**	1.287	0.012 (0.847)	0.033 (0.363)
COM	−2.452**	−4.054**	2.248	0.030 (0.489)	0.072 (0.572)
ELA	−1.856*	−2.879	5.347	0.014 (0.771)	0.070 (0.446)
FEN	−1,725**	−4.587**	0.688	0.235 (0.007**)	0.024 (1.000)
KOR	−1.798*	−12.458**	2.984	0.003 (0.588)	0.029 (0.660)
KOT	−1.768*	−5.625**	2.125	0.002 (0.757)	0.031 (0.417)
ORI	−1.312	−6.374**	0.622	0.016 (0.585)	0.051 (0.674)
TRI	−0.158	−2.215	4.148	0.036 (0.018*)	0.062 (0.032*)
EBU	−2.217**	−26.325**	1.368	0.008 (0.805)	0.082 (0.518)
ERI	−2.158**	−8.118**	1.648	0.125 (0.022*)	0.045 (0.946)
LYC	−2.345**	−15.741**	2.328	0.009 (0.771)	0.065 (0.525)
REU	−2.846**	−26.358**	1.447	0.006 (0.747)	0.025 (0.693)
URU	−2.251**	−26.222**	1.259	0.002 (0.867)	0.048 (0.872)
ARA	−1.489*	−2.748**	1.329	0.003 (0.364)	0.032 (0.699)
GLA	−1.675*	−26.697**	1.253	0.041 (0.215)	0.054 (0.639)
HAU	−1.477	−2.254	1.114	0.011 (0.124)	0.065 (0.413)
PAB	−0.347	−2.325	1.118	0.018 (0.806)	0.034 (0.362)
SCO	−2.449**	−2.118	1.985	0.023 (0.0425)	0.074 (0.804)

Time since the population expansion (t), Sum of square deviations (SSD) and its p-value (PSSD) for test of the validity of the sudden expansion model, Harpending’s Raggedness index (Raggedness) and its p-value (Pr) for the test of goodness-of-fit. For details on population see Table 1. *Significant at *P* < 0.05; **Significant at *P* < 0.01.

RETRACTED

**Figure 4:** Observed pairwise differences and expected mismatch distribution. Observed pairwise differences (bars) and expected mismatch distribution (solid line) under the sudden expansion model for (**A**) the Euamygdalus section, (**B**) Spartioides section, and (**C**) Lycioides section calculated for all of marker data.

## Discussion

Different PCR-based molecular markers were used for the assessment of wild almond species including RAPD and ISSR^33^, microsatellites^29, 33^ and AFLP^34^. In this study, three molecular marker methods (IRAP, REMAP, and S-SAP), based on insertion polymorphisms of Ty1-*copia* and Ty3-*gypsy* RTs were evaluated and compared to the AFLP, ISSR, SSR and SNP systems. We used a wide range of statistics to evaluate the performance of these molecular marker systems, including a measure of genetic polymorphism, the efficiency of polymorphism detection, and the capacity of different techniques to identify genetic relationships of accessions.

Of the 22 LTR primers investigated (Supplementary Table S5), Ty1-*copia*F and Ty3-*gypsy* F primers were designed to amplify products including the LTR of *copia* and *gypsy* retrotransposon-created IRAP fragments. The IRAP, REMAP, and S-SAP marker systems allowed the differentiation of all *Prunus* species analysed, as did the AFLP, ISSR and SSR systems. The dendrogram obtained from the REMAP similarity matrix (Fig. 3) appeared to be the most representative of the effective relationship between all accessions of wild almond species populations. In the REMAP phylogenetic tree, all *Prunus* species of different sections are in separate clusters^6, 34^. The EUA and LYC accessions were the most different, and the rest of the accessions were divided into two sub-clusters.

RETRACTED

The high reliability of the REMAP tree is most likely associated with the large-scale alterations in the genome induced by transposable elements. By comparison, SSR and, to some extent, AFLP (and other markers based on DNA digestion) essentially distinguish single nucleotide changes, which are affected by homoplasy and are bi-directional because the number of bands increase or reduce reversibly, so that it is difficult to infer valid phylogenetic connections of distantly related accessions^12, 15, 34^.

The ISSR phylogenetic tree was similar to the REMAP tree (results not shown). In this tree, it was also possible to differentiate the accessions of wild almond species that belonged to EUA and LYC, although LYC was positioned between the EUA and SPA groups and not into a sub-cluster of the EUA and LYC species, as in the REMAP tree. The similarity between REMAP and ISSR trees is strongly supported by the fact that they showed the highest value of correlation between cophenetic matrices and between similarity matrices (*r* = 0.970 and *r* = 0.952, respectively; Table 5) of all the dendrograms. Furthermore, various polymorphic bands, PIC, MI and SI values (Table 6) and the CV trends were similar in both of these molecular marker systems. The accuracy of REMAP and ISSR trees is shown by the higher bootstrap values than those characteristic for other dendrograms: bootstrap values are significant for the majority of the clusters (Fig. 3).

**Table 5:** Correlations between cophenetic matrices (above diagonal) and similarity matrices (below diagonal) obtained with different markers systems. Bold typeset indicates statistically significant (*P* ≤ 0.05) values.

	AFLP	IRAP	ISSR	REMAP	SSAP	SSR
**AFLP**	1	0.287	0.147	0.152	0.064	0.354
**IRAP**	0.3888	1	**0.358**	**0.458**	0.068	0.068
**ISSR**	0.2798	0.614	1	0.987	**0.048**	0.128
**REMAP**	0.2608	**0.548**	**0.987**	1	0.038	0.258
**SSAP**	0.6178	0.354	0.415	0.548	1	0.139
**SSR**	**0.4618**	0.154	0.048	0.098	0.042	1

**Table 6:** Summary of the average genetic diversity parameters in *Prunus* species determined using a subset of the most efficient 7 REMAP, 4 ISSR, 7 SSAP, 2 AFLP and 32 SSR markers.

Primer combinations	Total number of bands	No. of polymorphic bands	% of polymorphic bands	Shannon’s index (SI)	Marker index (MI)	Polymorphic information content (PIC)	No. of unique bands
REMAP	30.86b	19.86b	63.87b	0.57b	10.40b	0.50bc	12.29b
ISSR	34.75b	19.75b	55.85b	0.59c	9.37c	0.46c	9.00b
SSAP	62.29a	51.50a	80.19a	0.56a	22.63a	0.48a	25.33b
AFLP	77.50b	59.50b	76.77b	0.58b	23.75b	0.43b	18.00c
SSR	257b	257b	100b	3.91a	22.47b	0.87b	28b

Different letters represent statistically different values for *p* ≤ 0.05 (Duncan test).

RETRACTED

A Unique value not submitted to analysis of variance.

In the AFLP, IRAP, SSAP and SSR dendrograms, the sections of Euamygdalus and Lycioides species are not clearly separated from other species. Furthermore, the topology of each dendrogram is very different from the others and these differences are confirmed by low correlation values between cophenetic matrices and between similarity matrices (Table 5). Moreover, bootstrap values of the dendrograms are much lower compared to the REMAP and ISSR trees, and the SSR marker system required the highest number of bands to obtain a 10% CV and showed the lowest SI, MI and PIC values (Table 6). The unpredictability of the SSR dendrogram may be due to the use of the binary matrix in scoring SSR data. However, a dendrogram achieved by combining all marker systems data was very similar to that based on the binary matrix constructed from each marker (Fig. 5).

**Figure 5:** Heatmapobtained with the similarity simple matching (SM) coefficient pair group method with the arithmetical average clustering algorithm from all markers for 389 wild almond species. Bar graphs showing genetic diversity structure for 389accessions of *Prunus* species as assessed using STRUCTURE software. Each group is represented by a different color (blue, red and green).

Retro-transposons are mobile genetic elements that replicate by reverse transcription, which contributes to the physical size of the host genome. Retro-transposons are ubiquitous and abundant, which has played a major function in the structure and evolution of the plant genome. Retro-elements are long and cause a large-scale genetic alteration at the point of insertion, so insertions of variable numbers and sizes of retro-transposons into the host genome results in detectable polymorphisms. Previous studies have shown that Ty-1 *copia*-like-retrotransposons occurred in plant genomes in the early stages of evolution, and had diverged into heterogeneous subgroups before modern plant orders arose. There is clear evidence that retro-elements in the *Prunus* genome are heterogeneous because of their variable number and size. Analysis of the repetitive fraction of the peach genome showed that LTR retrotransposons comprise 18.56% of the genome, with 8.6% of Ty1-*copia*.Ty-1 *copia*-like-retrotransposon is also present in the *Citrus* genome at approximately 1.8–7.2 × 10^5^ molecules, and accounts for almost 17% of the genome. The IRAP and REMAP techniques are retrotransposon-based markers that are extensively used in plant breeding including genotyping and gene mapping^12, 35^.

RETRACTED

In the present study, the IRAP and REMAP banding patterns of the genotypes demonstrated a high level of polymorphism. In total, IRAP and REMAP analysis generated 93 scorable amplification products ranging from 250 to 2,000 bp. Of all the bands, 79 were polymorphic, with an average of 15 polymorphic bands per primer combination. The level of polymorphism was 84%, which was comparable between IRAP and REMAP.REMAP bands were polymorphic with all of the microsatellite primers investigated, and bands were not produced by amplification between microsatellite repeats (ISSR). The ISSR pattern established considerably less variation among wild almond species. The analysis of the genetic relationship of 389 wild accessions of almond showed that *Prunus* species are noticeably differentiated.

This is the first report of IRAP- and REMAP-based evaluation of *Prunus* and other RTN activity and genetic diversity in wild almond species. Of the tested primers, 19 IRAP and 34 REMAP primers were shown to amplify visible banding patterns and applied to study the RTN activity and genetic diversity among 389 wild almond species. RTNs may be in corporate in two orientations into the genome, and hence, any two members of one or more RTN families could be found head-to-head, tail-to-tail, or head-to-tail^12, 18^. Moreover, different RTN families may be integrated in each other. Therefore, in order to increase the likelihood of finding bands, we also combined primers from LTR end of different RTN families. A number of investigations have confirmed that primers based on LTR sequences of RTN families can be readily used across species, among closely related genera and even sometimes between plant families^12, 14^. In this study, single IRAP primers Tms1Ret1 and LORE1 and LORE2 created polymorphic banding patterns in the wild almond populations studied, showing the presence and movement of the aforementioned retro-elements in the *Prunus* species genome.

Madsen *et al*.^35^ reported that LORE1, a low-copy-number TY3-*gypsy* RTN family in the model legume species, *L. japonicus*, was active. LORE2A is estimated to be 600,000 years old, yet active in *L. japonicas* genome^36^. Tps12 may be inactive in the *Prunus* L. spp. genome as it creates a monomorphic banding pattern; nevertheless it produced greater polymorphism in combination with Tms1Ret1, representing the insertion of these two RTNs near or into each other in the *Prunus* genome. The primer based on Tps19 amplified no bands, representing its absence or fast divergence in *Prunus* species. Pearce *et al*.^37^ separated a large heterogeneous population of formerly uncharacterized Ty1-*copia* RTNs from pea (Tps) and demonstrated that each element group in pea is related to the more distantly-related *Vicia* species, demonstrating that heterogeneous populations of these elements were present throughout the evolution of the *Pisum* and *Vicia* genera from their common ancestor. It was shown that Tps12a and Tps19 have a high level of insertion polymorphism in pea and have been active during *Pisum* species evolution.

RETRACTED

Kalendar *et al*.^15^ showed the activity and insertion polymorphism of Bare1-based IRAP markers in *Hordeum*, *Triticum*, and *Aegilops* species. Tam *et al*.^38^, in a study of comparative analyses of genetic diversity in tomatoes, stated that RTN sequences isolated from one species can be used in related *Solanaceae* genera. REMAP amplification of the RTN families used indicated the insertion of the Tms1Ret1, as a native RTN, near the different SSRs in the *Prunus* genome. Non-native RTNs amplified bands in combination with a few SSR motifs, most likely signifying their low copy number, divergence, and preferential insertion within SSRs in *Prunus* L. spp. genome. The insertions of the RTN families in the vicinity of microsatellites have been formerly reported in barley and wheat^39^. Polymorphisms detected by markers based on non-native RTNs from *P. sativum* were low compared to those based on non-native RTNs from *L. japonicus*.

In total, 125 PCR amplicons designed from 100 EST contigs or genomic DNA that contained SNPs, INDELs and microsatellites were investigated using HRM based on the putative SNP information acquired from the almond and the *Prunus* EST databases. During sequencing of the HRM amplicon and flanking regions, 100 SNPs, as well as single nucleotide INDELs, were established in the population. HRM profiles of the fragments and evaluation techniques were established and the resulting SNP data were used to cluster the accessions of wild almond species. HRM is a novel, homogenous and closed-tube post-PCR method that can be applied to analyse the genetic variations as well as SNPs, polymorphism length and methylations of DNA in PCR amplicons^40, 41^. HRM requires an additional step, the melting process following cycling, and an additional reagent, a specific generic DNA fluorescence dye, to complete the assay compared to conventional PCR. Therefore, the time and costs of the analysis are similar to conventional PCR, but it omits the need for post-PCR separation required by many other assays. Therefore, an HRM assay has the advantages of speed, simplicity, and lower cost.

RETRACTED

HRM was intensively used for detecting mutations in known human genes. This approach for SNP analysis in plant species is very limited^42^. This study extended the application of the HRM method to the development of SNP markers by designing an HRM assay based on the putative SNPs from EST databases. This approach took advantage of the existing EST database, but avoided unnecessary sequencing efforts for putative SNPs in amplicons with in variant HRM curves in the test population. In our investigation, homozygous and heterozygous genotypes of all four SNP classes were distinguishable. In addition, the assay was able to resolve other variations, including INDELs, microsatellites, and complex multiple SNP amplicons.

As expected, the SNP frequencies were the lowest in coding regions (1:157), moderate in introns (1:130), and the highest in UTRs (1:51). These results are consistent with the findings in other taxa^43, 44^. The average ratio of transition-to-transversion was 1.84:1 in our analysis. Wu *et al*.^25^ reported a slightly lower value (1.16:1) in almond; however, the genome of other species was characterized by considerably higher values (e.g. 2.45:1 in humans^43^, and 1.53:1 in maize^44^). Transition bias over transversion has been fairly universal in the genome^45^, although differing results have been described in grasshopper pseudogenes^46^. Transition bias has been considered to be partially due to cytosine methylation^46^. Therefore, the low transition bias may reflect low methylation levels in the almond genome, and this could be significant because of the role of methylation in epigenetics and imprinting^41, 46^.

HRM has been applied in SNP detection, mainly in diagnosis and scanning for mutations in genes causing human diseases. We have shown this approach was valuable in the detection and recognition of plant SNPs. While many high-throughput SNP detection approaches, such as SNP microarrays, are cost-efficient for whole genome scanning in the species where genome-wide SNP information is available, it is expensive to assay the small amount of SNPs using these methods. It was demonstrated that HRM is a feasible means for this assay. As expanding DNA sequence information becomes available for species such as almond, HRM will be a valuable method for SNP detection and genotyping. This is particularly useful in plant cultivar identification, genetic mapping, QTL analysis, diagnosis of pathogenic species, and gene discovery. Furthermore, data from HRM analysis is portable, and therefore not only feasible for inter-genotype comparison, but also for library-based database construction. This feature may facilitate international collaborative efforts using SNP-based genotyping, and therefore genetics and biodiversity studies by using HRM analysis.

RETRACTED

Populations at demographic equilibrium or in decline present a multimodal distribution of pairwise differences, while populations that have experienced a sudden population expansion display a unimodal distribution^47, 48^. Tajima’s D and Fu’s Fs tests are expected to show significant negative values under population expansion and positive values under a population bottleneck and hence both of the parameters supported the sudden expansion of almond related species. In addition, growth in population size should result in elevated frequencies of rare alleles, explaining the unexpected 3–40% values found in the populations. It is also confirmed by the fact that most almond lineages differentiated during the Holocene^49^. Since wild almonds also have edible kernels human ancestors might have harvested their nuts as early as 780,000 years ago^50^. Therefore, it is reasonable to suppose that similarly to *P. dulcis* wild almond species were also influenced by human care.

## Methods

### Wild almond species and collecting regions

Wild almond species included in this study belong to the genus *Prunus*, subgenus *Amygdalus*, and were as follows: *P. carduchorum* (Bornm.) Neikle, *P. communis* (L.) Archang., *P. elaeagnifolia* (Spach) Fritsch, *P. fenzliana* Fritsch, *P. korschinskyi* Hand.-Mazz., *P. kotschyi* (Boiss. EtHohen.) Nab., *P. orientalis* Mill. (syn. *P. argentea* Lam.) and *P. trichamygdalus* Hand.-Mazz. in section *Euamygdalus* Spach; *P. eburnean* Spach, *P. Erioclada* Bornm., *P. Lycioides* Spach, *P*. *Reuteri* Boiss. Et Bushe and *P. Urumiensis* Bornm. in section Lycioides Spach; and *P. arabica* (Olivier) Neikle, *P. glauca* (Browicz) A.E. Murray, *P. haussknechtii* (C.K. Schneid.) Bornm., *P. Pabotii* Browicz and *P. Scoparia* Spach in section Spartioides Spach^6, 51, 52^. The number of accessions sampled per site varied from one to five, depending on the environment, diversity and accessibility at collection time^6^. A total of 389 accessions were sampled from the 18 studied species (Table 1).

The comprehensive procedure for field expeditions is presented in Sorkheh *et al*.^6^. Sites were selected based on literature^6^, indigenous information, or conspicuous presence. Collections were made from both wild and cultivated habitats, which were concentrated in two different regions in Iran. The first region (Azerbaijan and Kurdistan) is characterized by a relatively lush environment, a high biological diversity, and relatively under-developed agricultural activity. The second region (Shahrekord and Shiraz) is in a more xerophytic region with widespread agriculture (Supplementary Table S6; Fig. 6). Sampling sites and their geographic locations are reported in Table 1. The distance between samples was 200 m; the pairwise distance between the main regions was 100–500 km. Sampling was determined following the natural distribution of wild almond species in Iran, according to Sorkheh *et al*.^6^ in the wild. For the locations (see Table 1 for details), a specific agreement was not necessary because these locations are exterior-kept areas, and leaf gathering did not correspond to a threat to the sampled individuals. The sampled stands were selected to most closely represent the natural environment of the region. Collected leaves were stored at −80 °C until DNA isolation.

RETRACTED

**Figure 6:** Geographical locations of the wild almond species populations collected in Iran using ArcGIS for Desktop v10.4.

### Isolation of genomic DNA

DNA was isolated from the leaf tissue, using a modified CTAB method reported previously by Sorkheh *et al*.^6, 34^.

### IRAP analysis

A total of 22single and 60 IRAP primer combinations were used for evaluating RTN activity and for analyzing the genetic diversity in 389 individual wild almond species. Primers were designed based on RTN families isolated from *Prunus* species, *Lotus japonicus* and *Pisum sativum*: Tms1Ret1^16^ from *M. sativa*; LORE1^37^ and LORE2^16^ from *L. japonicus*; and Tps12a and Tps19^53^ from *P. sativum* (Supplementary Table S6). PCR amplification was carried out in a Bio-Rad thermocycler (Bio-Rad Laboratories Inc., Hercules, CA, USA). The PCR amplification profile was set according to Abdollahi Mandoulakani *et al*.^18^ with minor modifications^34^.

### REMAP analysis

For PCR, the amplification profile for REMAP markers followed those provided by Abdollahi Mandoulakani *et al*.^13, 50^ with minor modifications, as previously described by Sorkheh *et al*.^34^. A total of 48 REMAP primer combinations, derived from four single IRAP primers based on RTNs (Tms1Ret1, LORE2, LORE1, and Tps12a) with 19 inter simple sequence repeat (ISSR) primers A7, A12, B1, 438, 443, 459, 818, 825, 840, 848, 849, 857, A13, UBC815, UBC818, UBC825, UBC840, UBC848, and UBC857 were tested on four individuals of wild almond species to choose the primer combinations that would provide scorable and noticeable banding patterns. The annealing temperature of REMAP primer combinations depended on the primers (Table 2). In REMAP analysis, each LTR primer was used in combination with all 3′-anchored ISSR primers (Supplementary Table S5). PCR reactions and product staining were carried out based on the methods of Abdollahi Mandoulakani *et al*.^13, 54^ with minor modifications^34^.

RETRACTED

### ISSR analysis

For ISSR amplification using A7, A12, B1, 438, 443, 459, 818, 825, 840, 848, 849, 857, A13, UBC815, UBC818, UBC825, UBC840, UBC848 and UBC857 primers, only a single primer was utilized in each PCR reaction. Details of the PCR amplification are described by Abdollahi Mandoulakani *et al*.^13^.

### AFLP analysis

AFLP analysis was performed according to Sorkheh *et al*.^34^.

### S-SAP analysis

SSAP analyses were carried out following the same protocol, as summarized by Sorkheh *et al*.^34^, although 5′-end 6-FAM fluorophore-labelledCORTa, CORTb, GyRTa, GyRTb, GyRT1, GYRT3, and GYRT4 primers were used, in combination with M36 and M40 primers, which correspond to *Mse*I plus three extra selective nucleotides^34^. SSAP products were detected using an ABI 310 sequencer (Applied Biosystems, Foster City, USA).

### SSR and EST-SSR analysis

A set of 32 SSRs and 187 (12 of that were previously described, and 175 were developed in this study) EST-SSR primer pairs were selected based on previous information and new EST-SSRs were developed after database research (Supplementary Table S7 and Supplementary Table S8) on different *Prunus* species and identifying 33, 7, 2, 1 and 1 SSRs in peach, almond, plum, sweet cherry and sour cherry EST sequences, respectively (Supplementary Table S9). This set of markers was primarily displayed to confirm amplification in the collected samples of *Prunus* species, and afterwards 25 SSR and 9 EST-SSR primer pairs, covering eight linkage groups (G1 to G8), were chosen for subsequent analysis (MWG, Biotech, Germany). The forward primers were labelled with either 6-FAM or HEX fluorescent dye for recognition in a capillary genetic analyser. PCR reactions were carried out in a 96-well block cycler (BioRad Ltd. USA), in a final volume of 10 µl consisting of 10x PCR Buffer (Takara, Japan), 0.5 µM of each primer pair, 0.05 mM of each dNTP (Cina clone. Co., Iran), one Unit of *Taq* DNA polymerase (Takara, Japan), and 1 µl (100 ng) of genomic DNA. Cycling conditions were 94 °C for 3 min; 40 cycles at 94 °C for 0.5 min, 50–62 °C for 0.5 min, and 72 °C for 1 min, followed by 20 min at 72 °C for the final extension. Details are given by Rahemi *et al*.^29^.

### Discovery of the SNP markers

All EST (111,699) sequences of *Prunus* species including peach (*P. persica*; 80,797), apricot (*P. armeniaca*; 15,105), sweet cherry (*P. avium*; 6,035), Japanese apricot (*P. mume*; 4,589), almond (*P. dulcis*; 3,864), sour cherry (*P. cerasus*; 1,255) and European plum (*P. domestica*; 54) were downloaded from GenBank (ftp://ncbi.nlm.nih.gov/genbank/genomes/). To construct longer and less redundant sequences, publicly accessible ESTs were assembled from CAP3. Details of SNPs were preferred for HRM analysis, which were made available according to Wu *et al*.^25^ and Koepce *et al*.^55^.

RETRACTED

Forward and reverse primers on both sides of at least one assumed SNP were considered for HRM analysis using Primer 3^56^. Primer pairs were designed to have an annealing temperature of 60 ± 1 °C and to give an anticipated product size of 60–100 bp with few exclusions (Supplementary Table S3). Primers were analysed using NetPrimer to distinguish possible secondary structures, i.e. primer dimers, hairpins, palindromes and repeats (http://www.premierbiosoft.com/netprimer/netprimer.html, Premier Biosoft International, Palo Alto, CA), as secondary structures of primers are thought to influence the PCR amplification efficiency and, as a result, HRM accuracy. Secondary construction of the amplicons was analysed using the DINAMelt Server (http://www.bioinfo.rpi.edu/applications/hybrid/twostate-fold.php). The amplicons were considered suitable for HRM analysis when the DG value of the considered secondary structure was >−1 (Corbett Research 2006). The method for SNP detection and primer design is described in Wu *et al*.^25^, Koepke *et al*.^55^, and Salazar *et al*.^57^.

HRM analysis was based on the procedure of Wu *et al*.^25^, updated for the wild almond species. Briefly, PCR amplification was carried out in a total volume of 10 µL on an ABI Step one® and Step one Plus® real-time PCR Thermocycler (Life Technology, USA). The reaction mixture contained 40 ng almond genomic DNA, 10x PCR buffer, 1.5 mM MgCl_2_, 0.2 mM dNTP, 200 nM forward and reverse primers, 1.5 µM SYTO® Green-Fluorescent Nucleic Acid Stains(Molecular Probes™ by Life Technologies), and 0.6 U Takara *Taq* DNA polymerase (Takara, Co., Japan). Touchdown PCR has been previously described by Wu *et al*.^25^. HRM curve analysis was performed using the HRM module of the Real-Time PCR System Software (Life Technologies, USA). The melting data were standardized by correcting the initiate and stop fluorescence signals of all samples analysed for the same levels, according to Wu *et al*.^25^. Genotypes of the individuals were scored automatically by the software and verified manually. Whilst microsatellite polymorphism was involved in an amplicon, PCR products were separated using an 8% polyacrylamide (Cinagen Co, Iran) gel and stained with silver nitrate (Scharlau, Ltd. Spain). Details are provided by Sorkheh *et al*.^34^.

### Data analysis

The amplified fragments were achieved separately, equal to 1 or 0 for their occurrence or absence, respectively, and the acquired binary data were utilized for analysis. Each PCR product represented a single locus, and Shannon’s index (SI), marker index (MI) and polymorphic information content (PIC) was calculated. The SI, according to Shannon and Weaver^58^ is defined as:where *p*_*i*_ is the frequency of the i^th^ band in the sample. This formula was considered using the PopGene software version 1.32^59^. The MI was calculated according to Powell *et al*.^60^ as the product of expected heterozygosity (He) and the effective multiplex ratio (E). The heterozygosity of a locus is defined as:

$${\rm{He}}=1-\sum {{\rm{pi}}}^{2}$$

where *p*_*i*_ is the frequency of the i^th^ allele (band).

RETRACTED

The effective multiplex ratio of a primer combination is defined as:

$${\rm{E}}={\rm{nP}}0.95$$

where n is the number of loci detected per primer combination and P0.95 is the percentage of polymorphic loci^60^. Heterozygosity and P0.95 were calculated using GDA 1.0 software^32^. The polymorphic information content is commonly used as a representation of the expected heterozygosity^60^. Details are provided by Botstein *et al*.^61^. For the SSR markers, we considered expected heterozygosity (He), observed heterozygosity (Ho), the frequency of null alleles and the probability of identity (PI) using the IDENTITY 1.0 software^62^.

The calculated parameters were subjected to analysis of variance using SPSS 12.0. Different binary matrices related to different assays were imported into the NTSYS-PC2.01a package^63^ for cluster analysis. Genetic similarity matrices between genotypes were determined based on the simple matching (SM) similarity index^64^ for dominant multi-locus markers (AFLP, IRAP, ISSR, REMAP, and S-SAP), using the SIMQUAL routine, and according to the Nei coefficient^65^ for codominant SSR markers, using the SIMGEND routine. Dendrograms were constructed using similarity coefficients by the UPGMA with the NTSYS-PC2.01a software package. Bootstrap analysis (1,000 replacements) was carried out using the WinBoot software^66^, and differences between dendrograms were evaluated on the basis of correlations between similarity matrices and between cophenetic matrices calculated from the Mantel matrix correspondence test^67^.

The coefficient of variation (CV) trend from 5 to 120 polymorphic bands was evaluated on Nei coefficient matrices for SSR markers and on dissimilarity coefficient (1-SM) matrices for multilocus markers. For every molecular marker system, the CV trend was determined three times for three independent sets of 1,000 bootstrap analyses performed with the Phylip package^68^ on three randomized matrices of presence/absence. The number of loci required to acquire a 10% CV was approximated and proposed to the analysis of variance using the SPSS 12.0 package.

RETRACTED

For each retrotransposon family (Ty1-*copia* and Ty3 -*gypsy*), the two LTR sequences of each element were collected from the *Prunus* genome and evaluated. The main diverse LTR pairs for each retrotransposon family were used to calculate the number of nucleotide replacements by Kimura’s two-parameter model^69^, and the corresponding insertion ages for the transposable elements were then estimated using the formula T = K/2r, where T is the time of insertion, K is the difference parameter and r is the means of substitution rate. For r, the average value (4.11 × 10^−9^ subs/site/year) of the two values reported for woody perennial plants by Kay *et al*.^70^ was used.

With the aim of partition, the total genetic variation between and within populations, the analysis of molecular variance (AMOVA), was approved based on IRAP, REMAP, AFLP, SSR, S-SAP and ISSR data using GenAlEx 6^71^. The number of loci, polymorphic loci (%), the number of alleles or loci with a frequency higher or the same as 5%, the number of private loci or alleles, the number of less common loci with a frequency lower or equal to 25% and 50%, the mean of heterozygosity^28^, Nm (Number of migrants between populations), and standard error of mean heterozygosity were also calculated for each population using GenAlEx 6 for AFLP, IRAP, ISSR, REMAP, SSAP and SSR data.

Principal component analysis (PCA) was used to easily visualize relationships among the individuals and determine optimum number of clusters. The EIGEN module was used to calculate Eigen values and two-dimensional plots based on the variance-covariance matrix calculated between each two pairs of the one hundred accessions of wild *Prunus* species. Population structure was analysed using a model-based approach, Bayesian method, in STRUCTURE ver.3.0 software^72^. Since dominant markers were used in this study, each class of the accessions of wild *Prunus* species was treated as a haploid allele^73^. Model-based cluster analysis was used to test the number of populations (K). The most appropriate K can be detected by which values of log Pr (X/K) reach plateaus after a major decrease. We used both approaches to estimate K. No admixture and correlated allele frequencies models were used. For each population (K), 1000 iteration and 1000 burn-in period options were used. For each number of K from 1 to 10, five independent calculations were performed, and likelihood values obtained from these 10 calculations were averaged for each K.

Inferences on demographic history were obtained by neutrality tests and mismatch distribution, based on all marker data. As for neutrality test, Tajima’s D test and Fu’s Fs test^74^ were calculated using Arlequin 3.5^75^ with 10,000permutations. Mismatch distribution was constructed for each geographic population to test a model of exponential population growth^76^. A goodness of fit test was performed to test the validity of the sudden expansion model, using a parametric bootstrap approach based on the sum of square deviations (SSD) between the observed and expected mismatch distributions. The raggedness index which measures the smoothness of the mismatch distribution was calculated for each distribution. The demographic expansion parameter (*t*) was calculated using Arlequin 3.5^75, 77^.

RETRACTED

## Electronic supplementary material

Supplementary Figures

Supplementary Tables
